The article "Interactive effects of increased temperature, elevated pCO2 and different nitrogen sources on the coccolithophore Gephyrocapsaoceanica" was retracted in 2020. Reasons: errors in the data; errors in the methods; errors in the results or conclusions.

# Interactive effects of increased temperature, elevated pCO_2_ and different nitrogen sources on the coccolithophore *Gephyrocapsaoceanica*

**DOI:** 10.1371/journal.pone.0235755

**Published:** 2020-07-10

**Authors:** Citong Niu, Guicai Du, Ronggui Li, Chao Wang

**Affiliations:** College of Life Sciences, Qingdao University, Qingdao, PR China; Texas A&M University at Galveston, UNITED STATES

## Abstract

As a widespread phytoplankton species, the coccolithophore *Gephyrocapsaoceanica* has a significant impact on the global biogeochemical cycle through calcium carbonate precipitation and photosynthesis. As global change continues, marine phytoplankton will experience alterations in multiple parameters, including temperature, pH, CO_2_, and nitrogen sources, and the interactive effects of these variables should be examined to understand how marine organisms will respond to global change. Here, we show that the specific growth rate of *G*. *oceanica* is reduced by elevated CO_2_ (1000 μatm) in ${NO}_{3}^{-}$-grown cells, while it is increased by high CO_2_ in ${NH}_{4}^{+}$-grown ones. This difference was related to intracellular metabolic regulation, with decreased cellular particulate organic carbon and particulate organic nitrogen (PON) content in the ${NO}_{3}^{-}$ and high CO_2_ condition compared to the low CO_2_ condition. In contrast, no significant difference was found between the high and low CO_2_ levels in ${NH}_{4}^{+}$ cultures (p > 0.05). The temperature increase from 20°C to 25°C increased the PON production rate, and the enhancement was more prominent in ${NH}_{4}^{+}$ cultures. Enhanced or inhibited particulate inorganic carbon production rate in cells supplied with ${NH}_{4}^{+}$ relative to ${NO}_{3}^{-}$ was observed, depending on the temperature and CO_2_ condition. These results suggest that a greater disruption of the organic carbon pump can be expected in response to the combined effects of increased ${NH}_{4}^{+}$/${NO}_{3}^{-}$ ratio, temperature, and CO_2_ level in the oceans of the future. Additional experiments conducted under nutrient limitation conditions are needed before we can extrapolate our findings to the global oceans.

## Introduction

Coccolithophores are unicellular phytoplankton belonging to Class Prymnesiophyceae [1, 2]. They represent a prominent marine phytoplankton functional group and contribute greatly to the carbon cycle [3]. In addition to fixing CO_2_ into organic compounds through photosynthesis, these unique eukaryotic microalgae can also form calcite scales (coccoliths) through calcification [4]. Although the ballasting of photosynthetic products by coccoliths can efficiently transport carbon from the photic zone, the calcification process is also a net source of CO_2_ to the environment [5, 6]. Shifting of the carbon to nitrogen ratio (C/N ratio) produced by marine primary producers is proposed to function powerfully to determine atmosphere-ocean carbon partitioning [7]. Therefore, the relative strength of photosynthesis and calcification and the C/Nratio have a significant impact on the global biogeochemical cycle.

As a result of human activity, the atmospheric CO_2_ concentration has increased from the pre-industrial era value of 280 ppm to a current value of about 400 ppm, and it is expected to increase further up to 1000 ppm by the year 2100 under a business-as-usual CO_2_ emission scenario [8]. This will cause the seawater pH to decrease to ~7.8, which is 0.3 units lower than today’s value, leading to acidification of the oceans [9]. The increased atmospheric CO_2_level, in combination with other greenhouse gases, will lead to 2.5–6.4°C warming of the global air temperature by the year 2100 [10]. Accordingly, the surface sea temperature will rise by 2–3°C [11]. Both ocean acidification (OA) and warming will have a significant impact on marine phytoplankton communities [12–14]. These ocean environmental changes may have individual or interactive effects on the physiology and biochemical composition of coccolithophores. The calcification and growth rates of *Emilianiahuxleyi*, the most widely distributed coccolithophore species, are usually decreased by OA, although their photosynthesis is enhanced by a corresponding increase in pCO_2_ [15–17]. Additionally, Langer et al. (2009) reported that the malformation of coccoliths in *E*. *huxleyi* RCC 1238 increased with a temperature increase from 20°C to 25°C [18]. A recent study demonstrated that increased temperature aggravated the negative impacts of OA on the morphology of *E*. *huxleyi* [19].

Although the effects of OA and warming on coccolithophores have been studied intensively for the past decade, most studies were conducted under conditions with ${NO}_{3}^{-}$ as the only nitrogen source. However, ${NH}_{4}^{+}$ concentration and the ${NH}_{4}^{+}$/${NO}_{3}^{-}$ ratio are expected to increase in the future [20, 21], due to a combination of decreased ${NH}_{4}^{+}$ oxidation rates and increased nitrogen fixation of nitrogen-fixing cyanobacteria under elevated CO_2_ and low pH [22, 23]. ${NH}_{4}^{+}$ and ${NO}_{3}^{-}$ have distinct assimilation and metabolic pathways [24]. Generally, the fully reduced ${NH}_{4}^{+}$ is preferentially taken up and assimilated compared to the fully oxidized form of nitrogen in ${NO}_{3}^{-}$ [2]. The energetic cost is higher with ${NO}_{3}^{-}$ as the nitrogen source relative to ${NH}_{4}^{+}$, because after uptake, ${NO}_{3}^{-}$ must first be reduced to ${NO}_{2}^{-}$ and then to ${NH}_{4}^{+}$ [25]. Consequently, cells grown on ${NH}_{4}^{+}$ may have faster growth rates compared to those grown on ${NO}_{3}^{-}$ [26, 27]. Furthermore, the regulation of ${NO}_{3}^{-}$ and ${NH}_{4}^{+}$ assimilation and metabolism are quite different under varying conditions. For example, temperature affects the enzymes associated with ${NH}_{4}^{+}$ and ${NO}_{3}^{-}$ metabolism differently in diatoms; as a result, the uptake of ${NO}_{3}^{-}$ is higher at lower temperatures while the uptake of ${NH}_{4}^{+}$ increases with increasing temperature [24].

Changes in the cell redox status may also strongly affect the calcification of coccolithophores. Lefebvre et al. (2012) reported the calcification of *E*. *huxleyi*was decreased under ${NH}_{4}^{+}$ assimilation and enhanced under ${NO}_{3}^{-}$ assimilation [28]. A possible reason for this phenomenon involves the different numbers of protons generated during nitrogen assimilation. Assimilation of ${NH}_{4}^{+}$ as the nitrogen source produces excess H^+^, whereas assimilation of ${NO}_{3}^{-}$ produces excess OH^−^[29]. The inorganic carbon substrate ${HCO}_{3}^{-}$ needs to be dissociated into ${CO}_{3}^{2-}$ and releases extra H^+^ during calcification. It is possible that those extra H^+^ neutralize the OH^−^ generated during ${NO}_{3}^{-}$ assimilation, thereby promoting calcification. Conversely, the excess H^+^ generated during ${NH}_{4}^{+}$ assimilation could reduce the internal conversion of ${HCO}_{3}^{-}$ to H^+^ and ${CO}_{3}^{2-}$.

Marine phytoplankton tend to be confronted with the acidification and warming of seawater and changes in ${NH}_{4}^{+}$/${NO}_{3}^{-}$ ratio concurrently. It has been increasingly recognized that the interactive impacts of these variables must be investigated to understand how marine organisms will respond to global change [30]. In this study, we chose the coccolithophore species *Gephyrocapsaoceanica* to investigate the interrelated effects of CO_2_, nitrogen sources, and temperature on growth and elemental compositions, as the effects of these variables have been examined individually but the interactions among these variables have yet to be studied in this organism. *G*.*oceanica*, together with *E*.*huxleyi*, represent the most abundant coccolithophore morphospecies. In comparison with the ubiquitous *E*. *huxleyi*, which frequently forms extensive “milky water” blooms in high latitude ecosystems, *G*. *oceanica* is restricted to tropical and subtropical waters, and it occasionally forms massive blooms in transitional coastal waters of the Pacific Ocean [31]. Despite *G*.*oceanica* playing an important biogeochemical role in the ocean, its physiological performance and calcification under future global change are poorly understood compared to *E*.*huxleyi*. Additionally, there are considerable interspecific variations in responses to environmental changes, thus the different responses to multiple stressors among species should be elucidated.

## Materials and methods

### Experimental setup

The *G*.*oceanica* strain NIES-1318 used in this study was obtained from the National Institute for Environmental Studies (NIES, Tsukuba, Japan), and it was originally isolated from the East China Sea. Triplicate cultures were grown in Aquil nutrients (phosphate, trace metals, and vitamins) enriched artificial seawater, and nitrogen was supplied as either 100 μmol L^−1^${NH}_{4}^{+}$ or as 100 μmol L^−1^${NO}_{3}^{-}$. Eight conditions representing a matrix of CO_2_ (400(LC) or 1000(HC) μatm), temperature (20 or 25°C), and nitrogen source (${NH}_{4}^{+}$ or ${NO}_{3}^{-}$) were established, andcultures were illuminated with a light intensity of 190 μmol m^−2^ s^−1^under a 12: 12 h light-dark regime. Present environmental conditions are 400 μatm CO_2_ and 20°C (close to the annual mean surface temperature where *G*.*oceanica* was isolated), and predicted ocean acidification and warming conditions are1000 μatm CO_2_ and 25°C [10]. *G*.*oceanica* was pre-acclimated with semi-continuous culture in the above conditions for about 10 generations to reach stable growth and then for another 10 generations before sampling. The different CO_2_ conditions were realized by pre-equilibrating seawater with target CO_2_ concentrations (using a commercial CO_2_Enrichlor CE-100B, Wuhan Ruihua Instrument & Equipment Ltd, Wuhan, China) and loading them into 1 L polycarbonate bottles that were completely filled with culture medium and tightly closed without any gas exchange between the atmosphere and the medium. CO_2_ partial pressure output of the Enrichlor was stable as determined by continuous monitoring with a CO_2_ detector (M170, VaisasaOyj, Vantaa, Finland). All cultures were semi-continuously implemented by transferring the old cultures (100–150 ml) to the freshly prepared medium every two days. The final cell density was kept lower than 10^5^ cells ml^−1^ to make the carbonate system stable (pH variation <0.05, Table 1), and pH was measured with a pH meter that was calibrated with standard National Bureau of Standards buffer. Other seawater carbonate system parameters were calculated by CO2SYS software using the known parameters of pCO_2_, salinity, pH, temperature and nutrient concentrations [32]. The dissociation equilibrium constants K_1_ and K_2_of carbonic acid were determined according to Roy et al. (1993), and those of boric acid were from Dickson (1990) [33, 34].

**Table 1:** Mean values of the seawater carbonate system parameters under LC (400 μatm) and HC (1000 μatm) at 20 and 25°C. The cell concentrations of all cultures were maintained below 10^5^ cells ml^-1^ and pH variations were <0.04 units.

	Treatment	pH_NBS_	DIC (μmol kg^−1^)	pCO_2_ (μatm)	HCO_3_^−^ (μmol kg^−1^)	CO_3_^2-^ (μmol kg^−1^)	Total alkalinity (μmol kg^−1^)
20°C	HC	7.81±0.01^a^	2149.2±57.3^a^	1000±40^a^	2032.5±52.8^a^	89.72±4.2^a^	2261.5±63.1^a^
	LC	8.15±0.01^b^	1962.8±26.7^b^	400±40^b^	1776.9±20.8^b^	171.23±3.7^b^	2214.42±31.1^a^
25°C	HC	7.83±0.01^a^	2056.2±27.2^a^	1000±40^a^	2175.9±24.1^a^	105.3±2.6^a^	2309.3±30.2^a^
	LC	8.19±0.01^b^	1855.6±47.1^b^	400±40^b^	1999.6±38.5^b^	203.1±8.2^b^	2298.2±57.1^a^

The superscripts represent significant difference between HC and LC (p<0.05).

### Growth rates and cell size

Samples were taken in the middle of the light period. The specific growth rate (μ) and cell volume were measured using a Z2 Coulter Counter (Beckman, Buckinghamshire, UK). μ was calculated following the equation: μ = (ln C1 –ln C_0_)/(t1 –t_0_), where*t*_0_ and *t*_1_ were the time of inoculation and sampling, *t*_1_−*t*_0_ was the number of days between inoculation and sampling, and *C*_0_ and *C*_1_ were the cell concentrations at times*t*_0_ and *t*_1,_ respectively. The particle counter also provides the cell size distribution, and the cell volumes were calculated taking into account the cells’ shape following Hillebrand et al. (1999) [35].

### Measurement of POC, PON, and PIC

Duplicate samples (200 ml) taken in the middle of the light period were filtered onto 25 mm precombusted (450°C for 6h) Whatman GF/F filters and stored at –20°C. For analysis, one of the duplicate filters for each treatment was fumed over HCl for 12 h to remove inorganic carbon and then dried overnight at 60°C. The other filter was dried overnight at 60°C directly. All filters were packed in tin cups and analyzed on a varioMicro cube (Elementar, Germany). Particulate inorganic carbon (PIC)was calculated as the difference between total particulate carbon(TPC) and particulate organic carbon(POC). The production rates of POC, particulate organic nitrogen (PON), and PIC were calculated as P = cellular POC, PON, or PIC content (pg cell^−1^) × specific growth rate μ (d^−1^).

### Data analysis

Before parametric tests were performed, data were tested for homogeneity of variance and normality. Three- and two-way analysis of variance (ANOVA) combined with a Duncan’s post hoc test were used to determine the interaction among nitrogen source, pCO_2_, and temperature or between two of these variables, respectively. One-way ANOVA was applied to determine differences between two levels of a factor. Significance levels were set at p<0.05.

## Results

### Growth rates and cell volume

In the ${NO}_{3}^{-}$ cultures, growth rates were significantly lower in HC-grown cells than in LC-grown ones (Fig 1A), and the values were reduced by 14% (p<0.01) and 9.2% (p<0.01) at 20°C and 25°C, respectively. In the ${NH}_{4}^{+}$ cultures, elevated CO_2_ level enhanced the growth rates by 15.5% (p<0.01) and 102.6% (p<0.01) at 20°C and 25°C, respectively (Fig 1B). An increase of 5°C in temperature generally resulted in higher growth rates, except for in the ${NH}_{4}^{+}$ LC treatment, which had lower growth rates at 25°C compared to at 20°C. The growth rates were significantly higher in the ${NO}_{3}^{-}$ treatments than in the ${NH}_{4}^{+}$ ones under the LC condition (p<0.01), but they did not differ significantly in the HC environment (p>0.05). There were significant interactions among all three variables for growth rates (p<0.01, Table 2).

**Fig 1:** Specific growth rate (a, b) and cell volume (c, d) in NO_3_^—^ and NH_4_^+^-grown cultures under HC (1000 μatm) and LC (400 μatm) at 20°C and 25°C. The values are the means and error bars are standard deviations for triplicate cultures at each treatment (p<0.05).

**Table 2:** Three-way ANOVA analyses of interactive effects among temperature (T), pCO_2_ (CO_2_), and nitrogen sources (N) on physiological performance of *Gephyrocapsaoceanic*a.

	T×N	T×CO_2_	N×CO_2_	T×N×CO_2_
	*p* (F)	*p* (F)	*p* (F)	*p* (F)
Growth rate	<0.001** (501.4)	<0.001** (197)	<0.001** (872.9)	<0.001** (158.9)
Cell size	<0.001** (27.8)	<0.001** (14.4)	<0.001** (28.5)	0.121 (2.68)
POC	<0.001** (88)	<0.001** (18.9)	<0.001** (141.4)	<0.01** (4, 5.155)
POC_pro_	<0.001** (31.7)	0.233 (1.54)	<0.001** (22.4)	<0.001** (31.5)
PON	<0.001** (531.2)	<0.001** (64.4)	<0.001** (428.4)	<0.01** (9.85)
PON_pro_	<0.001* (56.8)	0.773 (0.086)	0.124 (2.63)	<0.001** (50.8)
POC/PON	<0.001** (28.1)	<0.05* (5.6)	<0.001** (53.4)	<0.001** (20.8)
PIC	<0.001** (56.8)	0.183 (1.933)	0.118 (2.73)	0.961 (0.002)
PIC_pro_	<0.001* (29.2)	0.195 (1.83)	<0.05* (5.38)	<0.05* (7.89)
PIC/POC	<0.05* (6.1)	0.273 (1.289)	0.113 (2.805)	0.392 (0.773)

“*” and

“**” represent significance levels at p<0.05 and 0.01 respectively.

Cell size was enlarged by 23.5%–46.4% (p<0.05) under elevated temperature and by 13%–35.2% (p<0.05) when ${NO}_{3}^{-}$ was replaced by ${NH}_{4}^{+}$ asthe nitrogen source (Fig 1C and 1D). In contrast, elevated CO_2_ consistently reduced cell size by 4.3%–22.1% (p<0.05). On the whole, cell volume was smallest in the HC ${NO}_{3}^{-}$ cultures at 20°C and largest inthe LC ${NH}_{4}^{+}$ cultures at 25°C, with values of 74.1 and 138.8 μm^3^, respectively.

### POC and POC production rates

Cellular POC content did not differ significantly between the HC and LC treatments in the ${NO}_{3}^{-}$ cultures (p>0.05, Fig 2A), but it was significantly reduced by 29.2% (20°C, p<0.01) and 27.7% (25°C, p<0.01) by elevated CO_2_ in the ${NH}_{4}^{+}$ treatments (Fig 2B). Increasing temperature increased POC by 63.2% in the ${NO}_{3}^{-}$ cultures (p<0.01) andby about 2-fold in the ${NH}_{4}^{+}$ ones (p<0.01). Nitrogen source did not affect POC content in the HC 20°C treatment, but it significantly increased it in the ${NH}_{4}^{+}$ treatment relative to the ${NO}_{3}^{-}$ treatmentunder other conditions (p<0.01), with the largest increase (53.3%, p<0.01) in the LC 25°C treatment. POC production rate showed the same trend as that of cellular POC with respect to nitrogen source and temperature treatment (Fig 2C and 2D). Elevated CO_2_ decreased POC production rate by 13.4% (20°C ${NO}_{3}^{-}$), 15.4% (25°C ${NO}_{3}^{-}$), and 18.2% (20°C ${NH}_{4}^{+}$), respectively, but increased it by 9.7% in the25°C ${NH}_{4}^{+}$ treatment (p<0.05).

**Fig 2:** POC (a, b) and POC production rate (c, d) in NO_3_^—^ and NH_4_^+^-grown cultures under HC (1000 μatm) and LC (400 μatm) at 20°C and 25°C. The values are the means and error bars are standard deviations for triplicate cultures at each treatment (p<0.05).

### PON, PON production rate, and POC to PON ratio

Cellular PON content was around 0.14 pmol cell^−1^ in the HC treatment regardless of temperature and nitrogen source, and it was 29.6% higher (${NO}_{3}^{-}$ cultures, p<0.01, Fig 3A) and 39.5% lower (${NH}_{4}^{+}$ cultures, p<0.01, Fig 3B) in the HC treatment than in the LC treatment. Increasing temperature increased this value (1.9 pg cell^−1^) by a factor of 1.5 for ${NO}_{3}^{-}$ cultures cells both in the HC and LC treatments, and by a factor of 2.4 in the HC treatment for ${NH}_{4}^{+}$ cultures, which was further increased by 50% (p<0.01) in the LC treatment to a value of 0.49 pmol cell^−1^. PON production rate showed a similar trend among different treatments, except for ${NH}_{4}^{+}$ cultures at 25°C (Fig 3D), for which no significant difference between the HC and LC treatments was found.

**Fig 3:** PON (a, b), PON production rate (c, d) and POC/PON (e, f) in NO_3_^—^ and NH_4_^+^-grown cultures under HC (1000 μatm) and LC (400 μatm) at 20°C and 25°C. The values are the means and error bars are standard deviations for triplicate cultures at each treatment (p<0.05).

The POC to PON ratio (C/N) ranged between 7.5 and 12.9. In the ${NO}_{3}^{-}$ treatment, C/N was 10 in the HC 20°C treatment. The ratio increased to about 12 and did not differ significantly among the other three conditions (p>0.05, Fig 3E). In the ${NH}_{4}^{+}$ treatment, C/N also was 10 in the HC 20°C condition (Fig 3F), but it was about 8 in the other three conditions.

### PIC, PIC production rate, and PIC to POC ratio

Cellular PIC content was consistently lower in the HC treatment than in the LC treatment. Values were in the range of 28%to46%regardless of temperature and nitrogen source (Fig 4A and 4B). PIC was greater at 25°C than at 20°C, particularly in the ${NH}_{4}^{+}$ treatments, for which the values were 3.3 times higher and 2.4 times higher the HC and LC treatments, respectively (p<0.01). Nitrogen source only affected PIC at 25°C; at this temperature, PIC content was 1.6 times lower in the ${NO}_{3}^{-}$ cultures compared to the ${NH}_{4}^{+}$ cultures for both the HC and LC treatments. The PIC production rate showed a similar trend to that of cellular PIC content among different conditions. The exception was the 25°C ${NH}_{4}^{+}$ cultures, for which PIC production rate did not differ significantly between the HC and LC treatments (Fig 4C and 4D).

**Fig 4:** PIC (a, b), PIC production rate (c, d) and PIC/POC (e, f) in NO_3_^—^ and NH_4_^+^-grown cultures under HC (1000 μatm) and LC (400 μatm) at 20°C and 25°C. The values are the means and error bars are standard deviations for triplicate cultures at each treatment (p<0.05).

The PIC to POC ratio (PIC/POC) was highest in the 25°C ${NH}_{4}^{+}$ treatments (Fig 4F), and there was no significant difference between the HC and LC treatments. In the other conditions, PIC/POC was about 30% higher in the HC treatment than in the LC treatment (p<0.05).

## Discussion

Coccolithophoreshave gained considerable attention because of their important roles in global biochemical cycles. Many researchers focus on the potential impacts of elevated pCO_2_- induced ocean acidification and increasing temperature on the most cosmopolitan coccolithophore species, *E*.*huxleyi* and *G*. *oceanica* [15, 36]. Most studies demonstrated that coccolithophores growth, which is a proxy for microbial reproductive fitness, was inhibited by elevated CO_2_. In our study, increased CO_2_ resulted in a lower growth rate in ${NO}_{3}^{-}$ cultures, which is in line with previous findings, whereas high CO_2_ enhanced *G*.*oceanica*’s growthin ${NH}_{4}^{+}$ cultures. This discrepancy may be related to the prominent difference in intracellular metabolism between cells using ${NO}_{3}^{-}$ or ${NH}_{4}^{+}$ as the nitrogen source, which can be inferred from the different POC and PON contents under varying situations.

From a physiological point of view, the decline of pH and associated increase of CO_2_ availability under ocean acidification should affect primary producers differently, with the former demanding more energy to maintain intracellular homeostasis as a result of the acidity of seawater and the latter saving energy for inorganic carbon acquisition due to higher availability of CO_2_ and ${HCO}_{3}^{-}$ [37]. Therefore, effects of ocean acidification on algae growth may largely depend on the organisms’ species-specific energetics as well as the related physiological regulation, and their responses to elevated CO_2_ subsequently may be modulated by temperature, nitrogen sources, and other environmental factors. Results of our study suggest that *G*. *oceanica* might use its own specific strategy to balance energy-using and energy-generating processes with those of C- and N-acquisition and assimilation under different combinations of nitrogen sources and CO_2_ levels. The assimilation of carbon and that of nitrogen are linked in multiple metabolic pathways, thus nitrogen and carbon metabolites have a variety of “cross-talk” within the cell and mechanisms to regulate the flux of metabolites into the cell [24].*G*. *oceanica* growth showed different responses to increased CO_2_ level based on the nitrogen source used, and this may be due to the readjusted metabolism of carbon and nitrogen when ${NO}_{3}^{-}$ was replaced by ${NH}_{4}^{+}$. For example, the 20°C ${NH}_{4}^{+}$ treatment had lower POC and PON quotas under high CO_2_ compared to low CO_2_,whereas at this temperature the ${NO}_{3}^{-}$-grown cells had the same content of POC and PON at the two CO_2_ levels. This result suggested that when using ${NH}_{4}^{+}$ as thenitrogen source, ocean acidification tended to stimulate cell division rather than storage of organic compounds.

It has long been argued that ${NH}_{4}^{+}$ would allow marine primary producers to grow faster and synthesize more organic nitrogen and carbon, mainly due to the lower energy requirements for ${NH}_{4}^{+}$ assimilation in comparison to ${NO}_{3}^{-}$ assimilation [38]. However, this phenomenon is not universal across microalgae species [26, 27]. In our study, ${NH}_{4}^{+}$ only promoted *G*. *oceanica* PON production, whereas it had no obvious effect on POC production or even inhibited cell growth rates. Other studies have also reported that growth on ${NH}_{4}^{+}$ rather than ${NO}_{3}^{-}$ provided cells with a lower energetic advantage than expected. For example, in the diatom species *Thalassiosirapseudonana*, cells supplied with ${NO}_{3}^{-}$ had equal growth rates and nitrogen content, as well as greater carbon content, compared to cells provided with ${NH}_{4}^{+}$ [39]. Levasseur et al. (1993) also found that diatoms (*Chaetoceros* sp.) cultured with ${NO}_{3}^{-}$ and ${NH}_{4}^{+}$ had similar growth rates and nitrogenand carbon quotas [40].

With an increase of 5°C in temperature, cells in the ${NH}_{4}^{+}$ treatment significantly decreased their POC/PON ratio, whereas no change in the ratio was detected in the ${NO}_{3}^{-}$ cultures. The different influence of temperature on enzymes associated with ${NH}_{4}^{+}$ and ${NO}_{3}^{-}$ metabolism may be responsible for the discrepancy. Nitrate reductase activity is known to be inversely related to temperature, whereas glutamine synthetase-glutamate synthase activity has a positive relationship with temperature across the same range [41].Thus, assimilation of ${NH}_{4}^{+}$ should be higher at warmer temperatures, and indeed, ${NH}_{4}^{+}$ uptake byboth dinoflagellate-dominated and diatom-dominated natural communities showed a positive relationship with increasing temperature, whereas ${NO}_{3}^{-}$ uptake showed an inverse relationship [42]. Taken together, the regulation of ${NO}_{3}^{-}$ and ${NH}_{4}^{+}$ uptake and assimilation differ with respect to environmental situations, and this feature can influence microalgae assemblage dynamics.

Lefebvre et al. [28] demonstrated that calcification in *E*. *huxleyi* was reduced under ${NH}_{4}^{+}$ assimilation and enhanced under ${NO}_{3}^{-}$ assimilation [28]. Tong et al. (2016) observed a similar phenomenon in *G*. *oceanica* when ${NO}_{3}^{-}$ was replaced by ${NH}_{4}^{+}$ as the nitrogen source [26]. They attributed this to the change in the redox status of the cell and the excess H^+^ generated during ${NH}_{4}^{+}$ assimilation. In our study, the *G*. *oceanica* PIC production rate (representing calcification rate) was decreased by ${NH}_{4}^{+}$ at 20°C, but the 25°C ${NH}_{4}^{+}$ cultures had a higher PIC production rate compared to the 25°C ${NO}_{3}^{-}$ treatment at the high CO_2_ level. This implies that the impact of different nitrogen sources on calcification can be altered by other environmental cues, and the underlying mechanism needs to be explored further. We conducted our experiments with a single species, and generating sufficient biomass to measure the different parameters required us to maintain the nutrient concentrations at levels much higher than those usually found in the open ocean. Thus, to extend our findings to the global carbon cycle, our experiments should be repeated with other coccolithophore species and under lower and more realistic oceanic nutrient concentrations.

In previous studies, the effects of seawater acidification and warming on coccolithophores have been extensively studied using ${NO}_{3}^{-}$ as the nitrogen source. Our results demonstrated that replacing ${NO}_{3}^{-}$ with ${NH}_{4}^{+}$ can greatly influence the combined effects of sea surface warming and future CO_2_ enrichment on *G*. *oceanica*. The positive effects of warming on the growth of coccolithophores under ${NO}_{3}^{-}$ conditions can transform into negative effects when cells are supplied with ${NH}_{4}^{+}$, but these effects can be alleviated by elevated CO_2_ concentrations. *G*. *oceanica* cells are grown at high growth and calcification rates under the combined conditions of elevated temperature, increased ${NH}_{4}^{+}$/${NO}_{3}^{-}$ ratio, and seawater acidification, which is the scenario predicted for future oceanic ecosystems. However, the responses of coccolithophores to environmental changes might depend on the timescale over which they are exposed, as longer exposure to changed conditions leads to different physiological responses [15].Therefore, caution should be exercised in directly extrapolating the results obtained from relatively short-term studies to long-term processes.
